The article "Effects of Electron Microscope Parameters and Sample Thickness on High Angle Annular Dark Field Imaging" was published in 2022. Journal: Scanning.

# Effects of Electron Microscope Parameters and Sample Thickness on High Angle Annular Dark Field Imaging

**DOI:** 10.1155/2022/8503314

**Published:** 2022-03-20

**Authors:** Pucheng Yang, Zheng Li, Yi Yang, Rui Li, Lufei Qin, Yunhao Zou

**Affiliations:** School of Materials Science and Engineering, Xiangtan University, Xiangtan, Hunan 411105, China

## Abstract

Scanning transmission electron microscopy (STEM) developed into a very important characterization tool for atomic analysis of crystalline specimens. High-angle annular dark field (HAADF) scanning transmission electron microscopy (STEM) has become one of the most powerful tools to visualize material structures at atomic resolution. However, the parameter of electron microscope and sample thickness is the important influence factors on HAADF-STEM imaging. The effect of convergence angle, spherical aberration, and defocus to HAADF imaging process has been analyzed through simulation. The applicability of two HAADF simulation software has been compared, and suggestions for their usage have been given.

## 1. Introduction

In recent years, dynamical diffraction is the major limitation to structure determination by electron methods, scanning transmission electron microscopy (STEM) which can effectively overcome this limitation by providing an incoherent image with electrons [1]. It has become a very popular and widespread technique and has been developed with different imaging modes (i.e., bright field (BF), annular bright field (ABF), and annular dark field (ADF)). High-resolution STEM using higher-angle scattered electrons (high-angle annular dark field, HAADF-STEM), where scattered electrons at higher angles are collected by an annular detector for STEM imaging, now attracts material scientists and semiconductor researchers [2] and becomes a powerful tool in characterizing nanoparticles [3, 4]), lithium ion batteries [5], quasicrystal [6–8], and alloy [9, 10]. HAADF has high resolution up to 40.5 pm [11, 12], image intuitive with the sensitive to chemical composition [13], and less damage to the sample, etc. It has become an important approach of material analysis at the atomic level due to the fact that its contrast depends highly on atomic number *Z* in a form of *Z*^*n*^ (*n* = 1.6–1.9) [14, 15].

There are two steps in STEM imaging: first, the parallel electron wave is emitted by the electron gun and converged by the lens to form the convergent electron wave; second, the convergent electron wave scans the surface of sample point by point, and each sample point will get an exit wave. The effect of imaging process in these steps should be considered: the influence of lens on image including the convergence angle [16], spherical aberration and defocus [17], and detector angle [18] and the influence of sample including the sample thickness and the atomic number [15, 19]. In STEM imaging mode, there are two theories that have been proposed to reveal the image formation process, such as multislice method [20, 21] and Bloch wave method [1, 22]. The Bloch wave method has the advantage of high calculation accuracy, but it can only suit for perfect crystal [23] and has a long calculation time [24, 25]. Compared to the Bloch wave method, the multislice method has the advantages of fast calculation speed and wide applicability [26]. However, the images calculated by the multislice method are greatly influenced by the thickness of slice [27]. Thus, it is important to choose an appropriate theory according to the requirement. In recent years, there are several approximation theories applied in simulated calculation for speeding up the STEM imaging, such as the frozen phonon model [28] and the absorptive potential approximation [29]. The frozen phonon model divides the wave function into an average and a fluctuating part, which is suitable for carrying out the incoherent averages [28]. And the absorptive potential approximation was proposed based on the fast Fourier transform (FFT) multislice approach [29].

The article "Effects of Electron Microscope Parameters and Sample Thickness on High Angle Annular Dark Field Imaging" was published in 2022. Journal: Scanning.

In general, HAADF provides incoherent images without any phase problem and can be directly inverted to object without additional image simulations [30, 31]. However, in a series of HAADF investigations [31–34] under STEM imaging condition, crystal tilt, probe convergence angle unavoidable factor (e.g., specimen thickness [35, 36], and collection angles of the detector [36], etc.) will impact on the quality of high resolution images. For example, sample bending and deviating slightly from the zone axis will result in remarkable contrast reduction and could cause atoms to be considerably displaced in HAADF image. Intensities of atomic-resolution HAADF images of zone-axis-oriented specimens change with defocus at rates that depend on lattice spacing, thickness, and strain which also effect on the intensities [27].

In this paper, the effect of electron microscope parameters and sample thickness on high angle annular dark field imaging was discussed in detail by simulation. In addition, simulation software QSTEM and Dr. Probe have been chosen for comparing their convenience in different simulation conditions.

## 2. The Frozen Phonon Model

In HAADF-STEM imaging, most of the signals received by annular detector come from phonon scattering [18].While frozen phonon model provides a simple method that the crystal potential is time-dependent under the assumption of independent atomic motion, under this assumption, the intensity of image *I*_*D*_ (*Z*) can be described as [37]

(1) $$\begin{array}{c} I_{D}\left(z\right)=\int_{0}^{z}\langle W^{2}\left(z^{\prime },t\right)\rangle {\left|\langle \psi \left(z^{\prime }\right)\rangle \right|}^{2}dz^{\prime }. \end{array}$$

The 〈*W*^2^(*z*′, *t*)〉 is related to the scattering factors, and the |〈*ψ*(z′)〉|^2^ is the elastic intensity. The image intensity is essentially obtained from the signal received by the detector. Under the screening of big angle annular detector in HAADF-STEM imaging mode, the final signal *g*(*x*_*p*_) from the probe position *x*_*p*_ should be

(2) $$\begin{array}{c} g\left(x_{p}\right)=\int {\left|\psi_{t}\left(k,x_{p}\right)\right|}^{2}D\left(k\right)d^{2}k, \end{array}$$

where the *ψ*_*t*_(*k*, *x*_*p*_) is the wave function diffracted onto the detector plane, and *D*(*k*) is the detector function [38].

(3) $$\begin{array}{c} D\left(k\right)=\begin{array}{cc} 1 & \text{for }k_{D_{\min}}\leq k\leq k_{D_{\max}}\\ 0 & \text{otherwise} \end{array}. \end{array}$$

The inner and outer angles of detector are the product of wavelength *λ* and the maximum and the minimum of the wave vector *k*. Therefore, *k*_*D*_max__and *k*_*D*_min__ are determined by the angle of detector. Thus, the key to analyze the intensity of HAADF image at the same detector angle is the exit wave function. While the exit wave function is the product of the incident wave function and sample transfer function which are determined by electron microscope and sample parameters, therefore, in the subsequent sections, we will analyze the effect of these parameters on HAADF image.

The article "Effects of Electron Microscope Parameters and Sample Thickness on High Angle Annular Dark Field Imaging" was published in 2022. Journal: Scanning.

## 3. Exit Wave

When the parameters of the incident electron beam and the sample are known, the equation of the exit wave can be obtained.

It started from the stationary Schrödinger equation:

(4) $$\begin{array}{c} -\frac{\hbar^{2}}{2\mu }\nabla^{2}\psi +U\psi =E\psi , \end{array}$$

where the *ψ* is the wave function, which presents the electron trajectory, *ћ* is the reduced Planck constant, *U* is the potential field function, *E* is the energy of the electron, and *μ* is the electron mass under relativistic correction. Due to the equation of wave-particle duality, *λ* = *h*/*p*, we know that *K*^2^ = 2meE/*h*^2^. Therefore, the Schrödinger equation can be written as

(5) $$\begin{array}{c} \nabla^{2}\psi \left(r\right)+4\pi^{2}K^{2}\psi \left(r\right)+4\pi^{2}U\left(r\right)\psi \left(r\right)=0. \end{array}$$

While under the condition of high energy approximate, the electron wave function can be written as the form of modulation wave:

(6) $$\begin{array}{c} \psi \left(r\right)=\phi \left(r\right)\exp\left(2\pi ik\cdot r\right). \end{array}$$

Substituting it into the Schrödinger equation, then

(7) $$\begin{array}{c} \Delta_{xy}\phi \left(r\right)+\frac{\partial^{2}}{\partial z^{2}}\phi \left(r\right)+4\pi {ik}_{xy}\nabla_{xy}\phi \left(r\right)+4\pi {ik}_{z}\frac{d\phi \left(r\right)}{dz}+4\pi^{2}U\left(r\right)\phi \left(r\right)=0. \end{array}$$

Under the condition of high energy approximate, (*∂*^2^/*∂z*^2^)*φ*(*r*) can be ignored, and we can obtain

(8) $$\begin{array}{c} \phi \left(r,z\right)=\exp\left\{\frac{iz}{4\pi k_{z}}\left[\Delta_{xy}+4\pi {ik}_{xy}\nabla_{xy}+4\pi^{2}U\right]\right\}\phi \left(r,0\right). \end{array}$$

Equation (8) shows that the relationship of the incident wave and the exit wave is determined by following factors: *z* is the sample thickness, *k*_*z*_ is the reciprocal of wavelength *λ*, Δ_*xy*_ is the direction of the scattering, and *U* is the crystal potential. These factors, effect on imaging process, will be analyzed in subsequent sections.

The article "Effects of Electron Microscope Parameters and Sample Thickness on High Angle Annular Dark Field Imaging" was published in 2022. Journal: Scanning.

## 4. The Effect of Electron Microscope Parameters on HAADF

In STEM imaging mode, the parallel electron waves from the electron gun pass through electron microscope before they are incident to the sample and become convergent electron waves. The incident waves will be affected by convergence angle, spherical aberration, and defocus. In order to illustrate the effects, BaTiO_3_ was taken as an example for simulation, and its structure model is shown in Figure 1. The simulation parameters are as follows: accelerating voltage is 300 kV (wavelength is 1.97 pm); the sample thickness is 82.7 Å, the tilt angle is 0, the convergence angle is 25 mrad, the spherical aberration and defocus are 0, and the detector angle is 50-250 mrad. The simulation software is QSTEM [39] which uses the frozen phonon model based on the multislice method [40].

### 4.1. Convergence Angle

When convergent electron waves are incident on the position *x*_*p*_ of the sample surface, the equation of incident wave function [38] is

(9) $$\begin{array}{c} \psi_{p}\left(x,x_{p}\right)=A_{p}\int_{0}^{k_{\max}}\exp\left[-i\chi \left(k\right)-2\pi ik\cdot \left(x-x_{p}\right)\right]d^{2}k. \end{array}$$

The *χ*(*k*) is the aberration function, *A*_*p*_ is the factor which comments ∫|*ψ*_*p*_(*x*, *x*_*p*_)|^2^*d*^2^*x* = 1, the influence of convergence angle on the incident wave function is the upper limit of integral *k*_max_ = *α*/*λ*, and *α* is the convergence semiangle.

As shown in Figure 2(a), when the convergence angle increases, the contrast of center atom Ti will decrease. It is more obviously in thick sample (i.e., Figure 2(b)). Besides, the spots of Ba atom are larger at small convergence angle, but smaller at large convergence angle. The same situations are obtained in reference [34] which analyzed the intensity profiles of 195 nm Si_0.8_Ge_0.2_ in different convergence angles. In the HAADF-STEM model, the electron probe with small convergence angle is more sensitive to crystal potential, the atomic brightness is larger, and the spot of atom is larger in small convergence angle.

The article "Effects of Electron Microscope Parameters and Sample Thickness on High Angle Annular Dark Field Imaging" was published in 2022. Journal: Scanning.

### 4.2. Spherical Aberration and Defocus

In fact, the spherical aberration of a real STEM is not 0. The convergence angle, spherical aberration, and defocus should be consider to choose the best condition for imaging [41, 42]. In Equation (9), *χ*(*k*) = *πλk*^2^(0.5*C*_*s*_*λ*^2^*k*^2^ − Δ*f*), it can be found that spherical aberration has a great influence on the incident convergent electron wave. In order to correct the influence of spherical aberration on the imaging process, the Scherzer focus condition [43] had been proposed. When the convergence angle is 10 mrad and spherical aberration is less than 0.1 mm, Figure 3(a) with the Scherzer focus condition has little changes as the spherical aberration increases. As shown in Figure 3(b), when defocus is 0, the simulated HAADF image becomes more and more anamorphose as the spherical aberration increases. When the convergence angle is 25 mrad, as shown in Figure 4, the anamorphose of the simulated HAADF images becomes worse as the spherical aberration is larger than 0.1 mm. It can be concluded that small convergence angle has good HAADF image at small spherical aberration conditions.

In HAADF-STEM mode, the Scherzer focus condition (Δ*f* = −1.15(*C*_*s*_*λ*)^0.5^) makes the transfer function have a wide flat area which leads to simulation images that have less abnormal structure information [17]. Therefore, it is obvious that the anamorphose deformation of the simulated HAADF images with the Scherzer condition is less than those who do not satisfy with it. And when the Scherzer focus condition is satisfied, the best convergence semiangle is

(10) $$\begin{array}{c} \alpha_{0}=1.41{\left(\frac{\lambda }{C_{s}}\right)}^{0.25}. \end{array}$$

Combined with the limit point resolution in STEM mode, *d*_0_ = 0.61*λ*/*α*_0_, it can be concluded that

(11) $$\begin{array}{c} d_{0}=0.43{C_{s}}^{0.25}\lambda^{0.75}. \end{array}$$

So, appropriate defocus and convergence angle should be chosen according to its spherical aberration. At present, the resolution of STEM image with spherical aberration correction has reached 40.5 pm [11]. Therefore, for an electron microscope with a certain spherical aberration, the key to high-quality STEM image is the appropriate defocus and convergence angle.

### 4.3. Detector Angle

In HAADF-STEM mode, the annular detector mainly receives high angle scattered electrons. Its scattering intensity can be expressed as the internal of inner angle *θ*_1_ to outer angle *θ*_2_ [18]:

(12) $$\begin{array}{c} \sigma_{\theta_{1},\theta 2}=\left(\frac{m}{m_{0}}\right)\frac{Z^{2}\lambda^{4}}{4\pi^{3}{a_{0}}^{2}}\left(\frac{1}{{\theta_{1}}^{2}+{\theta_{0}}^{2}}-\frac{1}{{\theta_{2}}^{2}+{\theta_{0}}^{2}}\right). \end{array}$$

In equation (12), *m* is the mass of high-velocity electrons, *m*_0_ is the static mass of electron, *Z* is the atomic number, *λ* is the wavelength, *α*_0_ is the Bohr radius, and *θ_0_* is the Born characteristic scattering angle.

The article "Effects of Electron Microscope Parameters and Sample Thickness on High Angle Annular Dark Field Imaging" was published in 2022. Journal: Scanning.

When the thickness of a sample is *t*, the intensity of exit electron wave is *I*, the number of atoms per unit volume is *N*, and the scattering intensity can be expressed as equation (13):

(13) $$\begin{array}{c} I_{s}=\sigma_{\theta_{1},\theta_{2}}\cdot NtI. \end{array}$$

Equation (12) can be transformed into equation (14):

(14) $$\begin{array}{c} \sigma_{\theta_{1},\theta 2}=\left(\frac{m}{m_{0}}\right)\frac{Z^{2}\lambda^{4}}{4\pi^{3}{a_{0}}^{2}}\left(\frac{{\theta_{2}}^{2}-{\theta_{1}}^{2}}{\left({\theta_{1}}^{2}+{\theta_{0}}^{2}\right)\left({\theta_{2}}^{2}+{\theta_{0}}^{2}\right)}\right). \end{array}$$

It obvious in Equation (14) that the larger inner angle *θ*_1_, the weaker the image intensity. The partial derivative of outer angle *θ*_2_ can be obtained:

(15) $$\begin{array}{c} \frac{\partial \sigma_{\theta_{1},\theta 2}}{\partial \theta_{2}}=\left(\frac{m}{m_{0}}\right)\frac{Z^{2}\lambda^{4}}{4\pi^{3}{a_{0}}^{2}}\left(\frac{2\theta_{2}}{{\left({\theta_{2}}^{2}+{\theta_{0}}^{2}\right)}^{2}}\right). \end{array}$$

The overall intensity of the image will be stronger with the increase of the outer angle. This also reflects that a larger detector angle range can obtain a stronger intensity image. However, the small inner angle may cause other signals to be detected (e.g., the diffraction contrast caused by Bragg reflection). Larger inner angle will also affect the relationship between the contrast of the atomic column and the atomic number *Z* in the final image which will be analyzed in the following sections. The intensity of the image atomic column is not simply linear with the sample thickness and the range of the detector angle [1]. Therefore, it is necessary to consider both the detector angle and image interpretation.

### 4.4. The Effect of Sample Thickness on HAADF

In imaging process, the incident wave is converged by the electron microscope and the surface of the sample is scanned point by point. There is no doubt that, sample parameters are also important influence on HAADF image. This section will discuss the influence of sample thickness on imaging process which is based on the simulation calculation of the multislice method.

The article "Effects of Electron Microscope Parameters and Sample Thickness on High Angle Annular Dark Field Imaging" was published in 2022. Journal: Scanning.

It can be found in Figure 5 that the contrast of center atoms (Ti) is stronger in thick sample. This phenomenon has been explained in [15]. Equation (12) shows that the intensity of atomic column is proportional to the square of the atomic number *Z*, while it should not consider the scattering intensity of one atomic array only in HAADF-STEM. For thin sample, if convergence semiangle *α*_0_ and the inner angle *θ*_1_ of the detector have the relationship:

(16) $$\begin{array}{c} \theta_{1}\geq 3\alpha_{0}, \end{array}$$

then the coherent effect between different atomic arrays of thin samples can be ignored. The approximation of the image intensity to the *n*-th power of the atomic number *Z* is very accurate. The range of *n* is 1.6-1.9 which is related to the inner and outer angle of detector.

## 5. Comparison HAADF Simulation Software

There is several software for HAADF simulation, and Dr. Probe and QSTEM are two free software which has wide used for researchers. In Dr. Probe software, the frozen-lattice approach [44] was used to simulate thermal-diffuse scattering (TDS). In this section, a horizontal comparison has been made between the two software to provide some reference for researchers. The simulation parameters of the two software are shown in Table 1.

### 5.1. Unit Cell with Small Size

PbTiO_3_ was chosen as the simulated material whose lattice constants are *a* = 3.90 Å, *b* = 3.90 Å, and *C* = 4.15 Å. As shown in Figure 6, the white highlights are Pb (*Z* = 82) atoms, and the gray and white ones are Ti atoms. The atomic number of O is too small which does not show in the image. Figure 6(c) is the structure projection of PbTiO_3_ at the [001] zone axis. The simulation results of the two software for small crystal cell have good quality, and both correctly reflect the crystal structure and atomic phase arrangement, while the contrast of Figure 6(b) is better. The contrast of Ti atoms in QSTEM is very fuzzy and difficult to distinguish. Moreover, the difference of the contrast and image point size of Pb atoms and Ti atoms in Figure 6(a) are too large. The image quality of Figure 6(a) is unnatural and unreal compared with Figure 6(b).

Figure 7 shows the simulated HAADF image of PbTiO_3_ along [001] at thicknesses with 40 unit cells. As shown in Figure 7(a), there are black dots in the center of the white bright spots representing Pb, but the contrast of Ti atom is improved obviously as compared with Figure 6(a). However, Figure 7(b) has problems in showing the contrast of Ti atoms, and it was difficult to observe the distribution of Ti atoms.

The article "Effects of Electron Microscope Parameters and Sample Thickness on High Angle Annular Dark Field Imaging" was published in 2022. Journal: Scanning.

### 5.2. Unit Cells with Moderate Size

MgAlO_4_ (*a* = *b* = *c* = 8.0858 Å) was chosen as the simulated material with moderate unit cell size whose lattice parameters are between PbTiO_3_ and Mg_44_Rh_7_. The thickness is 10 unit cells. The simulation results are shown in Figure 8. Compared with Figure 8(c), the white spots in Figure 8(a) and 8(b) represent Mg (*Z* = 12) atom. In Figure 8(a), the brightest atom is Mg atom, and the surrounding gray atom is Al atom. Due to the Mg atoms which are too close to the Al atoms in the projection of [001], the simulated image cannot distinguish them. Obviously, when unit cell has moderate size, QSTEM does better.

### 5.3. Unit Cell with Big Size

Mg_44_Rh_7_ (*a* = *b* = *c* = 20.148 Å) was chosen as the simulated material. The simulation results are shown in Figure 9. As shown in Figures 9(a) and 9(b), the white bright spots represent Rh (*Z* = 45) atoms, and the gray bright spots around the white bright spots represent Mg (*Z* = 12) atoms. Figure 9(c) is the projection structure model of Mg_44_Rh_7_ at the [001] zone axis. By comparing Figure 9(c), the simulated results of the two software are consistent with the projection crystal structure. However, there are differences in Mg atoms. Figure 9(b) can well display the contrast of Mg atoms, but Figure 8(a) is not obvious in showing the contrast of Mg atoms, and the contrast of Mg atoms among the four Rh atoms is insufficient.

### 5.4. Calculate Speed

In order to control variables, Dr. Probe and QSTEM were kept consistent during calculation, and single-core calculation was performed. QSTEM and Dr. Probe are used on the same PC. According to the simulation time records, the calculate time of the two software is shown in Table 2. QSTEM generally takes much longer time than Dr. Probe. In the simulation of small cell PbTiO_3_, the time of QSTEM was about 397% longer than that of Dr. Probe; in the simulation of medium cell MgAlO_4_, the time of QSTEM was about 164% longer than that of Dr. Probe; in the simulation of large cell Mg_44_Rh_7_, the time of QSTEM was about 440% longer than that of Dr. Probe. Therefore, Dr. Probe has higher computational efficiency than that of QSTEM.

## 6. Conclusion

With the development of scanning transmission electron microscopy, image interpretation in HAADF-STEM mode has become particularly important. In the imaging process, the influence of the electron microscope parameters and sample parameters must be considered. In this paper, the effect of electron microscope parameters and sample thickness on high angle annular dark field imaging were discussed in detail by simulation and experiment. In addition, simulation software QSTEM and Dr. Probe have been chosen for comparing their convenience in different simulation conditions. The conclusion is as follows:

1. Appropriate convergence angle is one of the key parameters for getting a good HAADF image. Small convergence angle has better image quality
2. Appropriate defocus and convergence angle should be chosen according to its spherical aberration
3. Under the condition of thin sample, sample thickness has little effect on HAADF image
4. QSTEM and Dr. Probe both are excellent like simulation software. Dr. Probe has higher computational efficiency than that of QSTEM

The article "Effects of Electron Microscope Parameters and Sample Thickness on High Angle Annular Dark Field Imaging" was published in 2022. Journal: Scanning.

## Figures and Tables

**Figure 1:** Projection structure model of BaTiO_3_: (a) at [001] direction and (b) at [011] direction.

**Figure 2:** Simulated HAADF image (the source size = 0.8 Å, detector angle = 50 mrad ~ 250 mrad, defocus = 0, spherical aberration = 0) and its intensity profile along the diagonal as the arrow shown of BaTiO_3_ at [001] axis zones with different convergence angles: (a) 42.3 Å thickness and (b) 82.7 Å thickness.

**Figure 3:** Simulated HAADF images (sample thickness = 82.7 Å, source size = 0.8 Å, detector angle = 50 mrad ~ 250 mrad, convergence angle = 10 mrad) with different spherical aberrations and defocus: (a) Scherzer focus condition and (b) defocus is 0.

**Figure 4:** Simulated HAADF images (sample thickness = 82.7 Å, source size = 0.8 Å, detector angle = 50 mrad ~ 250 mrad, convergence angle = 25 mrad) with different spherical aberrations and defocus: (a) Scherzer focus condition and (b) defocus is 0.

**Figure 5:** Simulated HAADF-STEM image (source size = 0.8 Å, detector angle = 50 mrad ~ 250 mrad, convergence angle = 25 mrad, defocus = 0, spherical aberration = 0) of BaTiO_3_ sample at different thicknesses and its intensity profile along the diagonal as the arrow shown.

**Figure 6:** Simulated HAADF-STEM images (sample thickness = 83.0 Å, source size = 0.8 Å, detector angle = 50 mrad ~ 250 mrad, convergence angle = 25 mrad, defocus = 0, spherical aberration = 0) along PbTiO_3_ [001]: (a) QSTEM, (b) Dr. Probe, and (c) structure model projection of PbTiO_3_ at the [001] zone axis.

**Figure 7:** Simulated HAADF-STEM images (sample thickness = 166.0 Å, source size = 0.8 Å, detector angle = 50 mrad ~ 250 mrad, convergence angle = 25 mrad, defocus = 0, spherical aberration = 0) along PbTiO_3_ [001]: (a) QSTEM and (b) Dr. Probe.

**Figure 8:** Simulated HAADF-STEM images (sample thickness = 80.9 Å, source size = 0.8 Å, detector angle = 50 mrad ~ 250 mrad, convergence angle = 25 mrad, defocus = 0, spherical aberration = 0) along MgAlO_4_ [001]: (a) QSTEM, (b) Dr. Probe, and (c) structure model projection of MgAlO_4_ at the [001] zone axis.

The article "Effects of Electron Microscope Parameters and Sample Thickness on High Angle Annular Dark Field Imaging" was published in 2022. Journal: Scanning.

**Figure 9:** Simulated HAADF-STEM images (sample thickness = 201.5 Å, s, detector angle = 50 mrad ~ 250 mrad, convergence angle = 25 mrad, defocus = 0, spherical aberration = 0) along Mg_44_Rh_7_ [001]: (a) QSTEM, (b) Dr. Probe, and (c) structure model projection of Mg_44_Rh_7_ at the [001] zone axis.

**Table 1:** The simulation parameters of QSTEM and Dr. Probe.

Parameters	QSTEM and Dr. Probe
Accelerating voltage	300 kV
Sources size	0.8 Å
Convergence angle	25 mrad
*C*_*c*_	1 mm
*C*_*s*_	0 mm
HADDF detector angle	50-250 mrad

**Table 2:** Simulate time of QSTEM and Dr. probe.

Crystal	QSTEM	Dr. Probe
PbTiO_3_	4641 s	934 s
MgAlO_4_	34443 s	13045 s
Mg_44_Rh_7_	204573 s	37861 s

## References

[1] Watanabe K., Yamazaki T., Hashimoto I., Shiojiri M. (2001). Atomic-resolution annular dark-field STEM image calculations. *Physical Review B Condensed Matter*.

[2] Sawada H., Tanaka N. (2014). Aberration correction in STEM(book chapter). *Scanning Transmission Electron Microscopy of Nanomaterials*.

[3] Chen Y., Chen Y., Qiu C., Chen C., Wang Z. (2015). HAADF STEM observation of the Au/CeO_2_ nanostructures. *Materials Letters*.

[4] Van A. S., Batenburg K. J., Rossell M. D., Erni R., Van Tendeloo G. (2011). Three-dimensional atomic imaging of crystalline nanoparticles. *Nature*.

[5] Tong Y. X., Zhang Q. H., Gu L. (2018). Scanning transmission electron microscopy: a review of high angle annular dark field and annular bright field imaging and applications in lithium-ion batteries. *Chinese Physics B*.

[6] Yang Z., Zhang L., Chisholm M. F., Zhou X., Ye H., Pennycook S. J. (2018). Precipitation of binary quasicrystals along dislocations. *Nature Communications*.

[7] Yasuhara A. J. P. M. (2015). The structure of an Al–Rh–Cu decagonal quasicrystal studied by spherical aberration (Cs)-corrected scanning transmission electron microscopy. *Philosophical Magazine*.

[8] Yubuta K., Yamamoto K., Yasuhara A., Hiraga K. (2014). Structure of an Al–Cu–Co decagonal quasicrystal studied by *C*s-corrected STEM. *Materials Transactions*.

[9] Duschek L., Kükelhan P., Beyer A. (2019). Composition determination of semiconductor alloys towards atomic accuracy by HAADF-STEM. *Ultramicroscopy*.

[10] Liu N., Zhang Z., Peng L., Ding W. (2015). Microstructure evolution and mechanical properties of Mg-Gd-Sm-Zr alloys. *Materials Science and Engineering: A*.

[11] Morishita S., Ishikawa R., Kohno Y., Sawada H., Shibata N., Ikuhara Y. (2018). Resolution achievement of 40.5 pm in scanning transmission electron microscopy using 300 kV microscope with delta corrector. *Microscopy and Microanalysis*.

The article "Effects of Electron Microscope Parameters and Sample Thickness on High Angle Annular Dark Field Imaging" was published in 2022. Journal: Scanning.

[12] Van A. S., Dekker A. J., Bos A., Van D. D. (2002). High-resolution electron microscopy: from imaging toward measuring. *IEEE Transactions on Instrumentation and Measurement*.

[13] Yasuhara A., Saito K., Nishijima M., Hiraga K. (2011). Characterization of Guinier-Preston zones in Mg-Gd-Zn alloys by using transmission electron microscopy. *Microscopy and Microanalysis*.

[14] Anderson S. C., Birkeland C. R., Anstis G. R., Cockayne D. (1997). An approach to quantitative compositional profiling at near-atomic resolution using high-angle annular dark field imaging. *Ultramicroscopy*.

[15] Hartel P., Rose H., Dinges C. (1996). Conditions and reasons for incoherent imaging in STEM. *Ultramicroscopy*.

[16] Weyland M. D., Muller D. A. (2005). Tuning the convergence angle for optimum STEM performance. *NanoSolutions*.

[17] Mory C., Colliex C., Cowley J. M. (1987). Optimum defocus for STEM imaging and microanalysis. *Ultramicroscopy*.

[18] Pennycook S. J., Berger S. D., Culbertson R. J. (1986). Elemental mapping with elastically scattered electrons. *Journal of Microscopy*.

[19] Liu Y., Zhu Y. L., Tang Y. L., Ma X. L. (2017). An effect of crystal tilt on the determination of ions displacements in perovskite oxides under BF/HAADF-STEM imaging mode. *Journal of Materials Research*.

[20] Dwyer C. (2010). Simulation of scanning transmission electron microscope images on desktop computers. *Ultramicroscopy*.

[21] Grillo V., Rossi F. (2013). STEM_CELL: a software tool for electron microscopy. Part 2 analysis of crystalline materials. *Ultramicroscopy*.

[22] Yamazaki T., Watanabe K., Kuramochi K., Hashimoto I. (2006). Extended dynamical HAADF STEM image simulation using the Bloch-wave method. *Acta Crystallographica*.

[23] Pennycook S. J., Jesson D. E. (1991). High-resolution incoherent imaging of crystals. *Physical Review Letters*.

[24] Yang Y., Cai C. Y., Yang Q. B. (2017). Comparison of two simulation methods in electron crystallography: BW method and a modified direct product method of scattering matrix. *Journal of Material Science & Technology*.

[25] Yang Y., Yang Q. B., Huang J. Y., Cai C. Y., Lin J. G. (2017). Quantitative comparison between real space and Bloch wave methods in image simulation. *Micron*.

[26] Nellist P. D., Pennycook S. J. (2000). The principles and interpretation of annular dark-field Z-contrast imaging. *Advances in imaging and electron physics*.

[27] Hillyard S., Silcox J. (1995). Detector geometry, thermal diffuse scattering and strain effects in ADF STEM imaging. *Ultramicroscopy*.

[28] Fanidis C., Dyck D. V., Landuyt J. V. (1992). Inelastic scattering of high-energy electrons in a crystal in thermal equilibrium with the environment I. Theoretical framework. *Ultramicroscopy*.

The article "Effects of Electron Microscope Parameters and Sample Thickness on High Angle Annular Dark Field Imaging" was published in 2022. Journal: Scanning.

[29] Ishizuka K. (2001). A practical approach for STEM image simulation based on the FFT multislice method. *Ultramicroscopy*.

[30] Pennycook S. J., Nellist P. D., Rickerby D. G., Valdrè G., Valdrè U. (1999). Z-contrast scanning transmission electron microscopy. *Impact of electron and scanning probe microscopy on materials research*.

[31] Yamazaki T., Kawasaki M., Watanabe K., Hashimoto I., Shiojiri M. (2002). Effect of small crystal tilt on atomic-resolution high-angle annular dark field STEM imaging. *Ultramicroscopy*.

[32] Cui J., Yao Y., Wang Y. G., Shen X., Yu R. C. (2017). Origin of atomic displacement in HAADF image of the tilted specimen. *Ultramicroscopy*.

[33] Kawasaki M., Yamazaki T., Sato S., Watanabe K., Shiojiri M. (2001). Atomic-scale quantitative elemental analysis of boundary layers in a SrTiO3ceramic condenser by high-angle annular dark-field electron microscopy. *Philosophical Magazine A*.

[34] Wu X., Robertson M. D., Kawasaki M., Baribeau J. M. (2012). Effects of small specimen tilt and probe convergence angle on ADF-STEM image contrast of Si_0.8_Ge_0.2_ epitaxial strained layers on (100) Si. *Ultramicroscopy*.

[35] Maccagnano-Zacher S. E., Mkhoyan K. A., Kirkland E. J., Silcox J. (2008). Effects of tilt on high-resolution ADF-STEM imaging. *Ultramicroscopy*.

[36] So Y., Kimoto K. (2012). Effect of specimen misalignment on local structure analysis using annular dark-field imaging. *Microscopy*.

[37] Van D. D. (2009). Is the frozen phonon model adequate to describe inelastic phonon scattering?. *Ultramicroscopy*.

[38] Kirkland E. J. (2010). *Advanced Computinging Electron Microscopy*.

[39] Koch C. (2002). *Determination of Core Structure Periodicity and Point Defect Density along Dislocations*.

[40] Cowley J. M., Moodie A. F. (1957). The scattering of electrons by atoms and crystals. I. a new theoretical approach. *Acta Crystallographica*.

[41] Hayani L. (2018). *Optimizing Precision of High-Angle Annular Dark Field Images in Scanning Transmission Electron Microscopy*.

[42] Kirkland E. J. (2011). On the optimum probe in aberration corrected ADF-STEM. *Ultramicroscopy*.

[43] Scherzer O. (1949). The theoretical resolution limit of the electron microscope. *Journal of Applied Physics*.

[44] Barthel J. (2018). Dr. Probe: a software for high-resolution STEM image simulation. *Ultramicroscopy*.

